# Psychometric Evaluation of the Narrow Corridor Walk Test (NCWT) on Advanced Walking Balance in People with Stroke

**DOI:** 10.1155/2022/1436715

**Published:** 2022-11-19

**Authors:** Longjun Ren, Tai Wa Liu, Shamay S. M. Ng

**Affiliations:** ^1^Department of Rehabilitation Sciences, The Hong Kong Polytechnic University, Kowloon, Hong Kong SAR, China; ^2^School of Nursing & Health Studies, Hong Kong Metropolitan University, Kowloon, Hong Kong SAR, China; ^3^Research Centre for Chinese Medicine Innovation, The Hong Kong Polytechnic University, Kowloon, Hong Kong SAR, China

## Abstract

**Objectives:**

To investigate (i) the interrater and test-retest reliabilities of completion time and number of steps in the Narrow Corridor Walking Test (NCWT); (ii) the minimal detectable changes (MDCs) in NCWT results; (iii) the correlations between NCWT results and stroke-specific outcome measures; and (iv) the optimal cut-off values of NCWT results for discriminating the difference in advanced balance ability between people with stroke and healthy older adults.

**Design:**

Cross-sectional.

**Subjects:**

Thirty people with stroke and 30 healthy older adults.

**Methods:**

People with stroke completed the NCWT on two separate days with a 7- to 10-day interval. The Fugl-Meyer Assessment (FMA), ankle dorsiflexor and plantarflexor muscle strength, Berg Balance Scale (BBS), Timed Up and Go (TUG) test, and the Chinese version of the Community Integration Measure (CIM) were used to assess. The healthy older adults completed the NCWT once.

**Results:**

The NCWT completion time and NCWT steps showed excellent interrater reliability and test-retest reliability and significant correlations with FMA, affected ankle dorsiflexor muscle strength, BBS score, and TUG completion time. A cut-off value of 7.40 s for NCWT completion time and 13.33 for the NCWT steps distinguished people with stroke from healthy older adults. The MDCs of the NCWT completion time and NCWT steps were 6.87 s and 5.50, respectively.

**Conclusion:**

The NCWT is a reliable clinical measurement tool for the assessment of advanced balance ability in people with stroke.

## 1. Introduction

People with stroke often have neurological impairment resulting in balance and mobility deficits and increased fall risk [1]. The fall incidence is 138 falls/10,000 patient-days [2] in people with stroke, which is approximately 5 to 29 times higher than that in healthy older adults [3]. Fall-related injuries can lead to immobility, loss of independence, and decreased quality of life [3], and one of the most serious fall-related injuries is hip fracture. The hip fracture rate of people with stroke is nearly 1.7-fold higher than that of healthy older adults, and falls are frequently reported during daily activities in restricted environments such as walking (23.9%), transferring (15.6%), and turning (18.3%), for which advanced balance ability is required. Indeed, previous studies reported that advanced balance ability measured by mediolateral stability during walking is a significant predictor of falls in people with stroke (odds ratio = 7.85) [4–6].

Several clinical measures have been widely adopted for assessing balance ability, such as the Berg Balance Scale (BBS) [7], Timed Up and Go (TUG) test [8], Tinetti's Performance-Oriented Assessment of Mobility (POAM) [9], and the Clinical Test of Sensory Interaction in Balance (CTSIB) [10]. However, these commonly used clinical measures are not without limitations. First, although the BBS has the benefit of assessing balance ability through a series of functional tasks, it has ceiling effects (24–35%), omits walking tasks, and focuses on the anticipatory balance ability instead of the necessitated actual response for maintaining balance in real life [11]. Second, the POAM and CTSIB are not sensitive enough to detect small progress or deterioration in balance ability [12], which reduces its clinical application value in real-life situations. Third, the TUG focuses on assessing turning and transferring ability, but there is little attention on walking, which is also an important aspect of advanced balance ability. These limitations highlight the need to develop a reliable and valid clinical measure that assesses advanced balance ability in restricted environments.

The Narrow Corridor Walking Test (NCWT) was originally developed by Kelly et al. to quantitatively assess the advanced balance ability of healthy older adults [13]. Using a three-dimensional motion analysis system, subjects are assessed while walking barefoot at normal speed within a 6 m narrow corridor [13]. The width of the corridor is normalized to 50% of the distance between the subjects' anterior superior iliac spines to standardize the challenge for subjects with different body shapes [13]. To transfer from laboratory-based assessment to clinical use, Gimmon et al. modified the NCWT by excluding laboratory-based equipment and related outcome measures such as step width and stride time [14]. The subjects are required to walk while wearing their own comfortable shoes, and the width of the shoe is added to the width of the narrow corridor; the advanced balance ability is assessed by the completion time, number of steps, step errors, and stumbles [14]. Although the NCWT has demonstrated sound psychometric properties in healthy older adults (good to excellent interrater reliability (intraclass correlation coefficient, ICC = 0.77 − 0.92) and weak to strong concurrent validity as measured by POAM (*r* = −0.22 to -0.62)) and in people with multiple sclerosis (MS) (poor to excellent rest-retest reliability (ICC = 0.18–0.94)), it has not been psychometrically examined in people with stroke.

People with stroke are in need of a clinical measure to assess advanced walking ability in real-life situations. Given the limitations of existing measures in assessing advanced balance ability and the unique test procedure of NCWT that simulates a real-life environment, it could be beneficial to extend the use of NCWT to the stroke population. Thus, the study aims of this study are to (i) determine the interrater and test-retest reliabilities of NCWT completion time and NCWT steps; (ii) identify the minimal detectable changes (MDCs) in the NCWT completion time and NCWT steps; (iii) investigate the correlations between the NCWT completion time and NCWT steps and stroke-specific outcome measures; and (iv) determine the optimal cut-off NCWT completion time and NCWT steps to discriminate performance between people with stroke and healthy older adults.

## 2. Methods

### 2.1. Sample Size Calculation

Referring to the reported good to excellent (ICC = 0.77 − 0.92) interrater reliability of NCWT results in healthy older adults [14], we assumed an excellent test-retest reliability (ICC = 0.90) of the NCWT completion time in people with stroke for sample size calculation. Thus, a minimum sample size of 26 was required to achieve 80% power and a 0.05 significance level for interrater reliability. As no previous study has investigated the correlation between the NCWT and stroke-specific measures used in the present study, we assumed moderate correlations (*r* = 0.50) between them. Thus, a minimum sample size of 21 was required to achieve 80% power at a 0.05 significance level. To draw a more reliable conclusion, the sample size was increased to 30.

### 2.2. Sample and Data Collection Procedure

The participants were recruited through poster advertisement in a local self-help network. The inclusion criteria for people with stroke were as follows: (i) an age over 50 years old; (ii) diagnosed with stroke at least 12 months before the study, and stroke type was confirmed by neurologist; (iii) ability to walk for 10 m independently with or without an assistive device; and (iv) sufficient cognitive function, with an Abbreviated Mental Test score ≥ 7 [15]. Participants with a history of neurological disease other than stroke or an unstable medical condition were excluded. The same criteria were applied for the recruitment of healthy older adults except that they did not have stroke.

All participants were invited to the university-based neurorehabilitation laboratory to complete all of the assessments. Ethical approval was obtained from the ethical committee of the local institution (HSEARS20160202006), and written informed consent was obtained from the participants before study initiation. For the stroke participants, the sociodemographic data sheet, Fugl-Meyer Assessment (FMA), ankle muscle strength test, Berg Balance Scale (BBS), TUG test, and the Chinese version of the Community Integration Measure (CIM) were administered on day 1 by rater A (Figure 1). The NCWT was assessed simultaneously by two raters (raters A and B). Then, the stroke participants were tested again on day 2 (7-10 days after day 1) by rater A. For the healthy older participants, only the sociodemographic data sheet and NCWT were administered on day 1 by rater A. This study was conducted in accordance with the Declaration of Helsinki [16].

### 2.3. Outcome Measurements

#### 2.3.1. NCWT

The NCWT was used to assess advanced balance ability in people with stroke [14]. During the test, subjects walked at a comfortable speed through a 6 m long narrow corridor formed by two carpets placed on flat ground (Figure 2). The width of the corridor was normalized to 50% of the distance between the subjects' anterior superior iliac spines plus the width of the plantar part of the shoe to ensure similar difficulty [14]. One practice trial before the test was allowed. The time through the corridor, number of steps, number of step errors, and number of stumbles in each trial were recorded. A step error was defined as contact of the participant's shoe with the carpet. A stumble was defined as the occurrence of imbalance in walking [17]. Each participant was required to perform three trials, and the mean was recorded. The NCWT completion time and steps have shown good test-retest reliability (ICC = 0.77 − 0.85) in healthy older adults [14]. As it is not practical and realistic to assess all NCWT parameters in people with stroke during routine assessment, we investigated the reliability of the NCWT completion time and steps in this study.

#### 2.3.2. FMA

The total FMA score is used to assess motor control including reflex, synergistic and isolated movements, and coordination in people with stroke [18]. It has shown excellent reliability (ICC = 0.83 − 1.00) in people with stroke [19].

#### 2.3.3. Ankle Muscle Strength

The Nicholas Handheld Dynamometer (Model 01160; Lafayette Instrument Company, Lafayette, IN, USA) was used to measure ankle muscle strength. The participants were in supine lying position with the hip and knee in zero degree flexion and ankle in the neutral position. The dynamometer was placed on the metatarsal heads on the dorsum and sole of the foot for ankle dorsiflexor and plantarflexor muscle strength measurement, respectively [20]. The participants were required to perform the maximal voluntary isometric contraction for 3 s. A resting interval of at least 1 min was set to eliminate the fatigue effect. The mean of three trials was recorded. This method has shown excellent test-retest reliability (ICC = 0.82 − 0.95) in people with stroke [21].

#### 2.3.4. BBS

The BBS was used to assess functional balance [7]. It has 14 functional tasks, with the total score ranging from 0 to 56 [7]. A higher score indicates better functional balance ability. It has shown excellent reliability (ICC = 0.95) in people with stroke [22].

#### 2.3.5. TUG Test

The TUG test was used to assess functional mobility [8]. In this test, the subject is instructed to perform a series of actions in sequence, which includes rising from a chair, walking 3 m, turning around, returning to the chair, and sitting down. Each subject is required to perform the TUG test three times, and the average completion time of the three trials is recorded [8]. A shorter TUG completion time indicates better functional mobility. This test has shown excellent reliability (ICC = 0.95) in people with stroke [8].

#### 2.3.6. CIM

The Chinese version of the CIM was used to assess community integration [23]. The CIM consists of 10 items [23]. The total score ranges from 10 to 50. Higher CIM scores indicate better community integration. In people with stroke, the CIM has demonstrated good internal consistency (Cronbach's *α* of 0.84) and good test-retest reliability (ICC = 0.84) [23].

### 2.4. Statistical Analyses

Statistical analyses were conducted with SPSS (version 26; IBM, Armonk, NY, USA). The Shapiro-Wilk test was used to examine the data normality. Differences in demographic and NCWT results between people with stroke and healthy older adults were examined using the independent *t*-test, Mann-Whitney *U* test, and chi-square test for parametric, nonparametric, and categorical variables, respectively. Interrater reliability was examined by ICC_3,2_ using the two-way mixed effects model, and each participant was assessed by two fixed independent raters. The test-retest reliability was examined by ICC_2,1_ using the two-way random effects model, and each participant was assessed by a randomly assigned rater from our research team [24]. ICCs > 0.90, 0.75–0.90, 0.50–0.75, and <0.50 indicated excellent, good, moderate, and poor correlation, respectively. The MDC at a 95% confidence interval was calculated with the equation $\text{Sx}\times \sqrt{2\left(1-r\right)}\times 1.96$, where Sx represents the standard deviation of the NCWT outcomes and *r* is the test-retest reliability coefficient. The standard error of measurement (SEM) was calculated using the equation $\text{Sx}\times \sqrt{1-r}$.

Correlations between the NCWT results and stroke-specific outcomes (FMA, affected and unaffected ankle plantarflexor and dorsiflexor muscle strength, BBS, TUG, and CIM) were calculated using Pearson's *r* and Spearman's rho for parametric and nonparametric variables, respectively. An “excellent,” “strong,” “moderate,” or “weak” relationship was indicated by a correlation coefficient of 1.00-0.90, 0.89-0.70, 0.69-0.40, or 0.39-0.10, respectively [25]. The significance level was set at *α* = 0.05. The Bonferroni correction was applied to adjust the significance level to *p* ≤ 0.006 (0.05/8) as there were eight stroke-specific outcomes in this study.

Receiver operating characteristic (ROC) curves were used to determine the cut-off values for differentiating the advanced balance ability of people with stroke and healthy older adults. Youden's index was used to identify the optimal cut-off values of the NCWT results with the trade-off between sensitivity and 1-specificity [24].

## 3. Results

### 3.1. Demographic Information of the Subjects

The demographic data of the people with stroke and healthy older adults are summarized in Table 1. There was a significant difference in sex between people with stroke and healthy older adults (*χ*^2^ = 6.944, *p* = 0.008).

### 3.2. NCWT Performance in People with Stroke and Healthy Older Adults

Table 2 summarizes the NCWT results and stroke-specific outcomes. People with stroke took a significantly longer time (15.93 ± 10.54 s) and more steps (18.6 ± 5.62) to complete the NCWT than the healthy older adults (5.82 ± 0.73 s and 10.96 ± 1.01, respectively).

### 3.3. Interrater Reliability, Test-Retest Reliability, and MDC

The NCWT completion time and steps showed excellent interrater reliability, as reflected by the ICC_3,2_ values of 1.000 and 0.987, respectively. Good to excellent test-retest reliability was also observed for the NCWT completion time and steps, as reflected by ICC_2,1_ value of 0.938 and 0.864, respectively (Table 3). The MDC and SEM are displayed in Table 3.

### 3.4. Correlation of NCWT Results with Other Outcome Measures

The NCWT completion time had a significant strong positive correlation (*r* = 0.793) with the TUG completion time and significant moderate negative correlations with the FMA score (*r* = −0.516), affected ankle dorsiflexor strength (*r* = −0.573), and BBS score (*r* = −0.545) (Table 4).

### 3.5. The ROC Curve of NCWT

The optimal cut-off NCWT completion time of 7.40 s (area under the curve (AUC) = 99.9%, sensitivity = 100.0%, and specificity = 99.7%; *p* < 0.001) and NCWT steps of 13.33 (AUC = 98.3%, sensitivity = 93.3%, and specificity = 100.0%) were identified as best to differentiate the advanced balance ability of people with stroke from that of healthy older adults (Figure 3 and Table 5).

## 4. Discussion

This was the first study to examine the psychometric properties of the NCWT in people with stroke. People with stroke took significantly longer and more steps to complete the NCWT than healthy older adults. The NCWT completion time and steps demonstrated good to excellent interrater and test-retest reliability. The MDCs of the NCWT completion time and steps were determined. The NCWT completion time was significantly correlated with the FMA score, affected ankle dorsiflexor strength, BBS score, and TUG completion time. The optimal cut-off completion time of 7.40 s and steps of 13.33 were identified as best to differentiate the advanced balance ability of people with stroke from that of healthy older adults.

### 4.1. NCWT Performance

This was the first study to examine the NCWT completion time (15.93 ± 10.54 s) and steps (18.60 ± 5.62) in people with stroke. Compared with the NCWT results from a previous study, people with multiple sclerosis (MS) outperformed those with stroke in our study on the NCWT with a shorter time (11.26 s) and less steps (13.28) [17]. This was because people with MS in the earlier study had higher levels of physical functioning. The age of people with MS was markedly younger than that of people with stroke in our study (32.6 vs. 61.53 years) [17], and the 2 min walking distance of people with MS was higher than that of people with stroke (174.52 vs. 103.24 m) [17, 26].

People with stroke in our study took a significantly longer time (mean difference: 10.11 s) and more steps (mean difference: 7.64) to complete the NCWT than healthy older adults. This finding is in line with a previous study, which reported that people with stroke had a lower walking speed than healthy older adults [27]. Loss of motor units [28], a decreased rate of motor unit firing rate [29], and altered neurophysiological properties of the motor unit [28] contribute to muscle weakness in people with stroke. In addition, impaired upper motor neurons disrupt corticospinal communication in stroke, which can result in muscle spasticity [30]. Therefore, muscle weakness and spasticity can contribute to the reduction of walking speed. Additionally, the physical limitations in people with stroke affect the kinematics of gait, causing gait dysfunction [31]. Such gait dysfunction includes step length asymmetry between the affected and nonaffected sides (asymmetry ratio = 0.18) and a smaller step length in people with stroke (52.7 ± 13.7 cm) than in healthy adults (75.5 ± 6.5 cm) [32], resulting in the former group taking more steps to complete the NCWT.

The difference in the NCWT completion time (10.11 s) and NCWT steps (7.64) between people with stroke and healthy older adults exceeded the MDC (6.87 s and 5.50, respectively), indicating that the between-group difference was a true difference and not a measurement error.

Two previous studies assessed the NCWT performance of community-dwelling elderly adults [14, 33]. The healthy older adults in our study (completion time: 5.82 s) outperformed those in previous studies (8.80-11.1 s) on the NCWT. Our healthy older population was relatively young (59.67 years) and none were fallers, whereas the subjects in previous studies were older (79.4-81.8 years) [14, 33], and 38.1% of the subjects were fallers in one study [33].

### 4.2. Reliability of the NCWT Results

In our study, the NCWT completion time and steps demonstrated good to excellent (ICC = 0.864 − 1.000) interrater and test-retest reliability in people with stroke. The key reasons for achieving excellent reliability were the standardized experiment protocol with clear instructions and the well-trained raters who conducted the NCWT assessment. The 7- to 10-day test-retest interval was optimal, as it was long enough to minimize the learning effect and short enough that no changes in the subjects' conditions occurred.

The interrater reliability of the NCWT completion time and steps of the current study (ICC = 1.000 and 0.987, respectively) was higher than that of a previous study in healthy older adults (ICC = 0.77 and 0.85, respectively) [14]. In our study, two raters recorded the completion time and steps simultaneously, whereas in the previous study, the subjects conducted NCWT twice on two different occasions within 1 hour and were assessed by two raters separately [14]. The increased variability in performance of the NCWT on two separate occasions resulted in a greater difference in the NCWT completion time and steps, which reduced the interrater reliability in the previous study of healthy older adults.

Compared with the test-retest reliability (ICC = 0.64 − 0.67) in people with MS [17], the NCWT completion time and steps showed a higher test-retest reliability (ICC = 0.864 − 0.938) in people with stroke of current study. In the previous study [17], the subjects with MS were required to complete the NCWT in both single-task and dual-task conditions on both day 1 and day 2. The variance of fatigue level among the subjects with MS may have contributed to the lower test-retest reliability [17]. By contrast, the subjects in our study only completed the NCWT in the single-task condition on day 1 and day 2. Therefore, the higher test-retest reliability in our study could be explained by controlling the factor of fatigue level.

### 4.3. Correlations between NCWT Results and Stroke-Specific Measurements

The NCWT completion time was moderately negatively correlated (*r* = −0.516, *p* = 0.004) with the FMA score but not the NCWT steps (*r* = −0.283, *p* = 0.136). A previous study [34] showed that the identification of less muscle synergy following stroke, which indicated better motor control, correlated with a better walking performance as measured by paretic limb propulsion in people with stroke. Barroso et al. found that the FMA-lower extremity score was significantly correlated (*r* = 0.678, *p* = 0.045) with paretic propulsion as measured by a gait motion capture system [35]. The NCWT assesses advanced balance and walking ability; thus, it was reasonable to identify a significant correlation between the FMA score and NCWT completion time. Gait dysfunction in people with stroke is characterized by reduced speed, step length, and asymmetry in temporal, spatial, kinematic, and kinetic gait variables [31]. The direction of step length asymmetry varies among individuals, with some participants exhibiting a shorter step length on the affected side and others exhibiting a shorter step length on the unaffected side [36]. The FMA scored on the performance of the affected side; thus, it was reasonable to find a nonsignificant correlation between the NCWT steps and FMA score.

The affected ankle dorsiflexor muscle strength was moderately correlated (*r* = −0.444, *p* = 0.001) with the NCWT completion time. To perform adequate foot clearance during the swing phase and to maintain eccentric contraction during the standing phase, sufficient muscle strength of the affected ankle dorsiflexor was required. The ankle dorsiflexor muscle strength is an independent predictor that explains 48.8% of the total variance of 6 min walking distance in people with stroke [37]. The weakness of the affected ankle dorsiflexor was shown to result in an increased swing time (healthy: 0.19 s and stroke: 0.40 s) and increased double support time (healthy: 0.38 s and stroke: 0.80 s) of the gait cycle [38], which eventually leads to a reduction in walking speed [39].

It was surprising to note that the affected ankle plantarflexor muscle strength was insignificantly correlated (*r* = −0.444, *p* = 0.014) with the NCWT completion time. The ankle plantarflexor provides forward power in the push-off phase and acts as a stabilizer in the standing phase of the gait cycle [37]. Studies have shown that walking speed is significantly correlated with ankle plantarflexor strength (*r* = 0.47 − 0.65) [40–42]. Our small sample size resulted in a nonsignificant correlation between the NCWT completion time and affected ankle plantarflexor strength. In fact, this correlation was significant before the Bonferroni correction (*p* = 0.006).

The BBS score was moderately correlated with the NCWT completion time (*r* = −0.545, *p* = 0.002) and steps (*r* = −0.419, *p* = 0.021). Both the BBS and NCWT assess balance ability during functional movement and use similar movement tasks. For example, the tandem task (item 8) in BBS requires the subject to place one foot directly in front of the other [7], whereas the NCWT requires the subject to walk and maintain the center of mass in a narrow corridor [14]. Both of those tasks demand excellent balance ability in the mediolateral direction [43, 44].

The TUG completion time was moderately to strongly correlated with the NCWT completion time (*r* = 0.793, *p* < 0.001) and steps (*r* = 0.494, *p* = 0.008). The TUG test consists of a series of tasks, including transfer and walking twice on a 3 m long track [8], and the NCWT is a walking task on a 6 m long narrow corridor [14]; thus, walking is a major component of both the NCWT and TUG. Furthermore, the NCWT results are correlated with a 2 min walking distance (*r* = −0.40 to -0.48) [17], and the TUG test completion time is correlated with walking speed (*r* = 0.84 − 0.92) [45]. Therefore, a correlation between the NCWT results and TUG completion time was expected.

There was a nonsignificant correlation between the NCWT completion time and CIM score (*r* = 0.089, *p* = 0.639). A previous study showed that functional impairments alone are insufficient to explain the variance of community integration [46]. The difference in measurement domains between the two measurements resulted in a nonsignificant correlation. The CIM measures community integration based on the subjects' self-reported feelings about social support, family relationship, environmental factors, and other factors [46]. In contrast, the NCWT is an objective measurement of advanced balance performance in walking, which may not reflect the subjects' feelings in a real-life situation. Thus, it was reasonable to find a nonsignificant correction between NCWT completion time and CIM score.

### 4.4. Optimal Cut-Off NCWT Completion Time and NCWT Steps

The NCWT completion time and NCWT steps showed an excellent ability to differentiate between people with stroke and healthy older adults in terms of advanced balance ability, with AUC values of 0.999 and 0.983, respectively. Thus, the NCWT completion time and NCWT steps had a probability of 99.9% and 98.3%, respectively, to correctly differentiate the advanced balance ability of people with stroke from that of healthy older adults. The optimal cut-off NCWT completion time (7.40 s) and NCWT steps (13.33) were much longer than the MDC of the NCWT completion time (6.87 s) and NCWT steps (5.50); thus, the optimal cut-off NCWT completion time and NCWT steps in this study detected a true difference between people with and without stroke rather than a measurement error.

### 4.5. Study Limitations

This study has several limitations. First, the NCWT assesses advanced balance ability while walking (e.g., completion time and number of steps) in a narrow corridor, but quantitative measurements of gait such as stride velocity, maximal excursion, and directional control were not included. Correlation analyses between the NCWT results and quantitative laboratory assessments of balance were not conducted. Future studies should use quantitative measurements to better understand advanced balance ability during walking. Second, the width of the narrow corridor was based on the subjects' pelvis width and shoe width; this setting does not mimic real-world situations in which walkways are of various widths. Future studies should consider assessing advanced balance ability in walkways of different widths. Third, the subjects were recruited from a local self-help community-dwelling group, and most of them had good recovery of motor function from stroke and were socially active. Thus, the generalizability of the results is limited to the population meeting our inclusion criteria. Fourth, our sample size calculation was not based on studies of people with stroke and was estimated using the excellent reliability and correlation in healthy older adults. Hence, the sample size may not have been large enough to determine a significant correlation between NCWT results and all other outcome measures in our study. A complementary study with a larger sample size is warranted. Lastly, this was a cross-sectional study, and we did not reveal any causal relationship.

## 5. Conclusion

The NCWT is a reliable and valid measurement to assess advanced balance ability during walking in people with stroke. The NWCT completion time was significantly correlated with the FMA score, affected ankle dorsiflexor muscle strength, BBS score, and TUG test completion time in people with stroke. The MDCs of the NCWT completion time and NCWT steps could reflect changes in advanced balance ability occurring over time, and the NCWT could differentiate advanced balance ability in people with stroke and healthy older adults. Moreover, the NCWT is easy to administer and only requires simple equipment and within 3-5 minutes to complete. It is a clinically relevant measure providing valuable information to plan for functional balance and gait training, particularly those trainings that target on mediolateral instability that is essential in maintaining balance when performing daily activities in restricted living environment.

## Figures and Tables

**Figure 1:** Flow chart of the assessment procedure. NCWT: Narrow Corridor Walking Test. ^∗^Stroke-specific assessments: FMA total: Fugl-Meyer Assessment total score; ankle muscle strength; BBS: Berg Balance Scale; TUG: Timed Up and Go test; CIM: Community Integration Measure.

**Figure 2:** Illustration of the Narrow Corridor Walking Test with an example of a step error. The white line in the middle is the narrow corridor formed by two carpets (gray blocks).

**Figure 3:** Receiver operating characteristic of the Narrow Corridor Walking Test (NCWT) completion time (a) and NCWT steps (b) for distinguishing the advanced balance ability of people with stroke from that of healthy older adults.

**Table 1:** Demographics.

	Stroke (*n* = 30)	Healthy (*n* = 30)	*p* value
Age (years)^†^	61.53 ± 6.74	59.67 ± 5.39	0.241
Sex (F/M)^‡^	13/17	23/7	0.008
Height (cm)^†^	161.95 ± 9.43	158.37 ± 9.71	0.153
Weight (kg)^†^	63.94 ± 11.90	58.38 ± 9.28	0.050
Body mass index (kg/m^2^)^†^	24.20 ± 3.73	23.37 ± 3.79	0.397
Poststroke duration (year)	3.14 ± 2.91		
Paretic side (L/R)	13/17		
Stroke nature (I/H/others)	11/17/2		

†: independent *t*-test; ‡: chi-square test; F: female; M: male; L: left; R: right; I: ischemic; H: hemorrhagic.

**Table 2:** NCWT outcomes and stroke-specific outcomes for people with stroke and healthy subjects.

	Stroke (*n* = 30)	Healthy (*n* = 30)	*p* value
Narrow Corridor Walking			
Time (s)^†^	15.93 ± 10.54	5.82 ± 0.73^∗^	<0.001
Steps (n)^†^	18.60 ± 5.62	10.96 ± 1.01^∗^	<0.001
Step errors (n)^†^	0.07 ± 0.20	0.00 ± 0.00	0.078
Stumbles (n)^†^	0.11 ± 0.25	0.03 ± 0.18	0.054
FMA	61.10 ± 21.46		
Ankle muscle strength (kg)			
Affected side			
Dorsiflexion	9.53 ± 5.87		
Plantarflexion	11.37 ± 5.33		
Unaffected side			
Dorsiflexion	16.65 ± 3.94		
Plantarflexion	15.96 ± 5.53		
BBS	50.20 ± 5.71		
TUG (second)	19.67 ± 8.49		
CIM	41.20 ± 6.70		

^∗^ *p* < 0.05. †: Mann-Whitney *U* test. BBS: Berg Balance Scale; CIM: Community Integration Measure; FMA total: Fugl-Meyer Assessment total score; TUG: Timed Up and Go test.

**Table 3:** Interrater and test-retest reliability, SEM, and MDC of NCWT results.

	Inter-rater ICC_3,2_ (95% CI)	*p* value	Test-retest ICC_2,1_ (95% CI)	*p* value	SEM	MDC
NCWT completion time	1.000 (1.000-1.000)^∗^	<0.001	0.938 (0.879-0.970)^∗^	<0.001	2.48	6.87
NCWT steps	0.987 (0.972-0.994)^∗^	<0.001	0.864 (0.734-0.933)^∗^	<0.001	1.98	5.50

^∗^ *p* < 0.05. CI: confidence interval; ICC: intraclass correlation coefficient; MDC: minimal detectable change; SEM: standard error of measurement.

**Table 4:** Correlations between NCWT results and other outcomes (all correlations are Spearman's rho).

	NCWT completion time	*p* value	NCWT steps	*p* value
FMA	Rho = −0.516^∗^	0.004	Rho = −0.283	0.136
Ankle muscle strength				
Affected side				
Dorsiflexor	Rho = −0.573^∗^	0.001	Rho = −0.219	0.245
Plantarflexor	Rho = −0.444	0.014	Rho = −0.167	0.377
Unaffected side				
Dorsiflexor	Rho = −0.277	0.138	Rho = −0.047	0.803
Plantarflexor	Rho = −0.216	0.252	Rho = −0.130	0.493
BBS	Rho = −0.545^∗^	0.002	Rho = −0.419	0.021
TUG	Rho = 0.793^∗^	<0.001	Rho = 0.494	0.008
CIM	Rho = 0.089	0.639	Rho = −0.130	0.495

^∗^After the Bonferroni correction, the significant level was adjusted to *p* < 0.05/8 = 0.006. BBS: Berg Balance Scale; CIM: Community Integration Measure; FMA total: Fugl-Meyer Assessment total score; TUG: Timed Up and Go test.

**Table 5:** Values of area under the receiver operating characteristic curve, sensitivity, and specificity for the optimal cut-offs of NCWT.

	Area under the curve	*p* value	Sensitivity (%)	Specificity (%)	Optimal cut-off
NCWT completion time	0.999^∗^	<0.001	100.0	99.7	7.40
NCWT steps	0.983^∗^	<0.001	93.3	100.0	13.33

^∗^ *p* < 0.05.

## Data Availability

The data that support the findings of this study are available on request from the corresponding author.
